# Photogrammetric Anthropometry to Determine the Female Waistline

**DOI:** 10.7759/cureus.21798

**Published:** 2022-01-31

**Authors:** Mohd Altaf Mir, Amborish Nath, Rajesh Maurya

**Affiliations:** 1 Burns and Plastic Surgery, All India Institute of Medical Sciences, Bathinda, Punjab, IND; 2 Plastic Surgery, Himalayan Institute of Medical Sciences, Dehradun, IND

**Keywords:** abdominoplasty, liposuction, waist-sculpting, female waist line, golden ratio

## Abstract

Background: In this study, we attempted to develop a reference guide to determine the female waistline based on the golden ratio for waist sculpting in females, which may help in waist sculpting by liposuction or non-invasive techniques.

Material and methods: To understand the anatomy of the waist, we studied the 60 photographs of females and measured the distances between important anatomical landmarks. The different values and proportions obtained were compared between different groups of heights and two groups of BMI using Statistical Package for the Social Sciences (SPSS) version 23 (IBM Corp., Armonk, NY) through analysis of variance (ANOVA).

Results: There is a golden ratio in the distances between xiphoid to waist and waist to the abdominal crease that is close to 1:1.66, and the waist is at the junction of the upper 2/5th and lower 3/5th of the height from xiphoid to abdominal crease. The location of the waist is at one-third of the whole length of the abdomen (the whole length of the abdomen being the length from the xiphoid to the pudendal cleft).

Conclusions: We observed in our study that there is a definite mathematical relationship between the length of the abdomen and the waist position, which may be applied for female waist sculpting.

## Introduction

Women all over the world, regardless of culture or ethnicity, want to possess an attractive waist. So, there is an increasing need to define the waist while performing liposuction procedures or non-invasive lipolysis and cool sculpting procedures [1]. Tummy tuck or abdominoplasty is the fifth most performed cosmetic surgery in the United States; 140,834 procedures were done in 2017 [1]. Liposuction and waist creation are done along with abdominoplasties to augment the beauty of the abdomen.

Non-invasive methods of body contouring are also being designed for body contouring [1,2]. There has been no literature until now defining the exact anatomical location of the waist. So, we embarked upon reviewing photographs of women considered standard and ideal and taking measurements to define the exact anatomical location of the site where the waist should be created. Similar studies have been done before using images available on the internet and from similar sources [3].

We present this report of our attempt to develop a reference guide based on different measurements, which is based on the more objective guidelines that may be applied for female waist sculpting.

## Materials and methods

Study design and settings

A cross-sectional study of photogrammetric anthropometry to determine the female waistline was done to develop a reference guide for waist sculpting in female waist sculpting by liposuction or by non-invasive techniques. The study has been done in accordance with the declaration of Helsinki version 2013. A hundred photographs of females of different ethnicities with known age, weight, height, hip, and waist size were selected from different online-published open-access fashion magazines for which consent is not required; however, the anonymity has been maintained. 

Photograph/sample selection

The photographs with diffuse lighting were not used as they obscured natural crease lines. Full frontal photographs without bend or torsion at the waist of the females of different ethnicities were chosen such that it had the abdominal crease line and the vulvar cleft exposed. Hundred out of 300 photographs of females of different ethnicities were selected and rated a score of 7 and more on a scale of 0 to 10 according to the choice of 10 females and 10 males not related to the medical profession. An expert panel was appointed to judge and select the photographs and to consider whether the photographs were aesthetically optimal (7 or more) on a scale of 0-10. The panel consisted of three independent plastic surgeons who rated the photographs from the above-selected pool of 100 photographs. The 70 photographs with the highest ratings (score of 7 and more) were selected. However, we had to decrease the number down to 60 after exclusion of the photographs with overtly bent back, with some minor twisting of the waist, and where the abdominal crease was not properly visible.

Photogrammetric anthropometry

Photogrammetric anthropometry was performed as shown in Figure 1 (Panels A and B) (authors' own creation). The distance from the upper end of the pudendal cleft to the umbilicus is “p.” The umbilicus is said to be lying in the midpoint between the upper end of the pudendal cleft and the xiphoid [4-7]. Measuring the distance of the pudendal cleft from the umbilicus provided us with the approximate location of the xiphoid process. The distance from the approximate area of the xiphoid process and the umbilicus “a” is equal to the distance from the upper end of the pudendal cleft to the umbilicus “p” (p = a). A natural crease line exists just above the mons pubis indicating the area where the recti muscles attach to the pubic bones. The distance from the umbilicus to the abdominal crease line “b” is marked. The abdominal crease line is prominent in most females; however, in skinny or athletic females, the crease is faintly conspicuous. A point “1” was selected on this crease line, where it intersects the line drawn between the umbilicus and the pudendal cleft. The waist is defined as the narrowest point of the torso below the ribs and above the hips. On the frontal images of the models, the waist points were marked on both the sides of the torso and joined by a line called waist point line “y,” and the point where this line intersects the line between the xiphoid and the umbilicus is chosen as the point “2.” The distance from the waist point line to the abdominal crease line, i.e., the distance between 1 and 2 is “x.” The following ratios a/b, a/x, b/y, and x/y were calculated.

**Figure 1:** Indirect anthropometry on photograph Figure 1A shows indirect anthropometry on the photograph of a female model, while Figure 1B shows indirect anthropometry on the pencil sketch of an ideal female model created by authors. Both panels show a vertical line from the xiphoid to upper end of the pudendal cleft. A lower transverse line passes through the lowest most point of the naturally existing abdominal crease line just above the mons pubis. This line intersects the vertical line at point 1. Another horizontal line is drawn at the narrowest point of the torso below the ribs and above the hips (waist). This line intersects with the vertical line at point 2. It also shows a, b, x, and y distances as described in the article.

Data collection and statistical analysis

The data collected were tabulated in a Microsoft Excel spreadsheet (Microsoft Corporation, New Mexico, USA) followed by statistical analysis. The different values and proportions obtained were compared between different groups of heights and two groups of BMI using Statistical Package for the Social Sciences (SPSS) version 23 (IBM Corp., Armonk, NY) through analysis of variance (ANOVA).

## Results

The mean age, weight, height, BMI, and waist to hip ratio calculated on photogrammetric anthropometry are 22.65 ± 2.84 years, 50.41 ± 4.85 kg, 167.38 ± 6.19 cm, 18.00 ± 1.56, and 0.71 ± 0.043, respectively. The calculation of different ratios as depicted in Figure 1 from the above measurements is depicted in Table 1 and the remaining figures in this article.

**Table 1:** Summary of different parameters and ratios calculated on photogrammetric anthropometry of 60 females to determine the ideal female waistline a, b, x, and y are described in Figure 1. IS, Insignificant.

Parameters	Height > 170 (cm)	Height ≤ 170 (cm)	BMI > 18.5 (kg/m^2^)	BMI ≤ 18.5 (kg/m^2^)	Statistics
Pencil art of models	29	31	28	32	-
Mean age (years)	22.05 ± 2.84	21.89 ± 2.73	23.67 ± 2.27	23.80 ± 2.50	p > 0.05 (IS)
Mean weight (kg)	51.41 ± 4.85	49.81 ± 4.05	50.41 ± 4.85	48.81 ± 4.95	p > 0.05 (IS)
Mean height (cm)	170.01 ± 6.19	169.88 ± 6.09	170.08 ± 6.29	169.98 ± 6.09	p > 0.05 (IS)
Mean BMI (kg/m^2^)	18.95 ± 1.56	18.09 ± 1.26	18.75 ± 1.66	18.09 ± 1.25	p > 0.05 (IS)
Mean hip to waist ratio	0.70 ± 0.09	0.71 ± 0.04	0.70 ± 0.08	0.71 ± 0.05	p > 0.05 (IS)
Mean a/b ratio	1.55 ± 0.15	1.54 ± 0.16	1.55 ± 0.17	1.54 ± 0.14	p > 0.05 (IS)
Mean a/x ratio	1.01 ± 0.06	1.02 ± 0.05	1.02 ± 0.06	1.03 ± 0.07	p > 0.05 (IS)
Mean b/y ratio	1.16 ± 0.25	1.15 ± 0.26	1.14 ± 0.26	1.14 ± 0.27	P > 0.05 (IS)
Mean x/y ratio	1.39 ± 0.29	1.41 ± 0.99	1.45 ± 0.19	1.46 ± 0.29	p > 0.05 (IS)

The mean a/b ratio calculated is 1.54 ± 0.14. Comparing the a/b values in different groups of heights, the P-value was found to be 0.997, which is an insignificant difference in value among the subgroups (Figure 2).

**Figure 2:** Box plot comparison of a/b values based on height It shows the comparison of the a/b values in different groups of heights and shows that there is an insignificant difference in value among the subgroups.

Comparing the a/b values in the two groups of BMI, the P-value was found to be 0.145, which is an insignificant difference in value among the subgroups (Figure 3).

**Figure 3:** Box plot comparison of a/b values based on BMI It shows the comparison of the a/b values in different groups of BMI and shows that there is an insignificant difference in value among the subgroups.

The mean a/x ratio calculated is 1.02 ± 0.06. Comparing the a/x values in different groups of heights, the P-value was found to be 0.997, which is an insignificant difference in value among the subgroups (Figure 4).

**Figure 4:** Box plot comparison of a/x values based on height It shows the comparison of the a/x values in different groups of heights and shows that there is an insignificant difference in value among the subgroups.

Comparing the a/x values in the two groups of BMI, the P-value was found to be 0.145, which is an insignificant difference in value among the subgroups (Figure 5).

**Figure 5:** Box plot comparison of a/x values based on BMI It shows the comparison of the a/x values in different groups of BMI and shows that there is an insignificant difference in value among the subgroups.

The mean b/y ratio calculated is 1.14 ± 0.26. Comparing the b/y values in different groups of heights, the P-value was found to be 0.967, which is an insignificant difference in value among the subgroups (Figure 6).

**Figure 6:** Box plot comparison of b/y values based on height It shows the comparison of the b/y values in different groups of heights and shows that there is an insignificant difference in value among the subgroups.

Comparing the b/y values in the two groups of BMI, the P-value was found to be 0.839, which is an insignificant difference in value among the subgroups (Figure 7).

**Figure 7:** Box plot comparison of b/y values based on BMI It shows the comparison of the b/y values in different groups of BMI and shows that there is an insignificant difference in value among the subgroups.

The mean x/y ratio calculated is 1.45 ± 0.19. Comparing the x/y values in different groups of heights, the P-value was found to be 0.730, which is an insignificant difference in value among the subgroups (Figure 8).

**Figure 8:** Box plot comparison of x/y values based on height It shows the comparison of the x/y values in different groups of heights and shows that there is an insignificant difference in value among the subgroups.

Comparing the x/y values in the two groups of BMI, the P-value was found to be 0.305, which is an insignificant difference in value among the subgroups (Figure 9).

**Figure 9:** Box plot comparison of x/y values based on BMI It shows the comparison of the x/y values in different groups of BMI and shows that there is an insignificant difference in value among the subgroups.

The above calculations show no significant differences among the various subgroups. So, we can assume that a = 1.5 b (since a/b is approximately 1.5) and (a + b)/a = 1.66. This shows that the distance “a” is roughly equal to the distance “x,” since a/x is roughly equal to 1. And b/y is roughly equal to 1, so the distance “y” is roughly equal to the distance “b.” Distance “a” bears a relationship with distance “b,” and “x” with “y,” and the two ratios of a/b are equal to x/y. There is a relationship between the distance “a” and the length of the abdomen “(a + b),” which is 1.66, equal to a near golden ratio. Similarly, the distance “x” bears a similar relation with the length of the abdomen “(x + y).”

## Discussion

A well-done tummy tuck when combined with liposuction can produce remarkable results. At times, the profile of the abdomen after abdominoplasty is flat on the sides, and it requires to be coupled with liposuction or other non-invasive procedure to create a waist [2]. There has been no objective anatomical guide to the location of the waist. Previously, the terms such as “just below the ribs” and “just above the navel” were used. There is no convincing textual lead available as yet.

We have used photographs of females, and similar techniques have been used before to study anthropometry [3]. It is easy and convenient to access photographs through the internet. We referred to a study by Lee et al. where the investigator studied the photographs of models and used software to alter the light exposure to define the xiphoid process [3]. It is difficult to clearly define the xiphoid process by that method; however, we can get an approximate idea about the location of the xiphoid process.

In our study, we manipulated the images by changing the light exposure using software to identify the abdominal crease. The pudendal or the labial cleft could be used as a reference landmark because the photographs selected had to have exposed labial cleft as a selection criterion. We have calculated the approximate supposed distance of the xiphoid from the navel using the knowledge from the previous studies about the abdominoplasties [4-7]. These studies mention the distance between the xiphoid to umbilicus and umbilicus to the pudendal cleft is the same. We have taken this guide in our study. There is a mention of the relation between the umbilicus and the position of the waist. The umbilicus is said to lie 1-4 cm below the waistline [4-7]. However, there is no defined landmark for the waist, with respect to the length of the abdomen. The distance of the navel from the waistline may vary among patients of different heights.

The subjects of the photographs used in the study were of age 22.65 ± 2.64 years, height of 167.38 ± 6.19 cm, and BMI of 18.0024 ± 1.566. There was no significant variation among the various parameters measured on the basis of height or BMI. The measurements were on females photographed in standing positions only. So, the effect of change of the measurements on lying down could not be commented upon. The abdominoplasty surgeries are done with the patient in a supine position, so the waist position of the patient in the supine position might be different from the position on standing. However, the marking for the procedure is always done in a standing position prior to the surgery for which our results would be helpful to predict the female waistline.

We found in our study that the waist bears a mathematical relation with the xiphoid process and the abdominal crease. The ratio y:x (= 1:1.5) suggests that the waist is at the junction of the upper 2/5th and lower 3/5th of the height from the xiphoid to the abdominal crease. Hence, the vertical distance between the xiphoid and the abdominal crease and the distance from the waist to the abdominal crease line bears a ratio of 1.66:1.

Abdominoplasty involves the transverse incision near the abdominal crease region; the scar is placed just 1-2 cm below the abdominal crease, roughly taken as 6-7 cm above the pudendal cleft as described in the textbook of Plastic Surgery by Peter C Neligan [8]. The abdominal crease region is chosen because it is also normally the region where the upper hemline of underwear rests and the scar can be hidden under the underwear or the swimwear. The scar aligns well with crease lines, hence is cosmetically favorable.

The relation of the umbilicus with the abdominal crease has never been studied before, and we also found that the umbilicus also has a mathematical relationship with the xiphoid and the abdominal crease. The distance from the xiphoid to the umbilicus is 1.5 times the distance from the umbilicus to the abdominal crease, and the vertical distance between the xiphoid and the abdominal crease and the distance between the xiphoid and the umbilicus have a ratio of 1.66:1, which is reasonably close to the golden ratio. The above knowledge can act as a guide while creating the neo-umbilicus during abdominoplasty as well.

Whole length of the abdomen from xiphoid to pudendal cleft “A” = a + b = 2a = 2 x 1.5b = 3b. The b is approximately equal to y. Hence A = 3y and y = A/3. So, we can say that the location of the waist in our selected population is at one-third of the whole length of the abdomen from the xiphoid process (the whole length of the abdomen being the length from the xiphoid to the pudendal cleft).

Thus, these anthropometric calculations may guide us about the approximate position of the waist for body contouring in females. Until now, the guidelines to the location of waste have been 1-4 cm above the navel as per plastic surgery textbook guidelines or just below the ribs as per finest art books. Some fine art books suggest that the level of the elbow with the arms by the side in a standing position is the level of the waist [9]. Thus, we could deduce the waist position based on bony landmarks. Hence the discrepancies due to considerations of the soft tissue landmarks can be sorted out. There are only a few studies for the description of waist localization [10-12], and hence, our study might add to the literature the indirect anthropometric evaluation of waist position in adult females.

We observed in our study that there is a definite mathematical relationship between the length of the abdomen and the position of the waist, which may be applied for female waist sculpting. However, a drawback of our study is the number of images studied was 60; a greater sample size could have given us more accuracy. Further studies of this kind may be needed for the augmentation of evidence, and studies with measurements directly on human subjects are also needed to validate the evidence. We are looking forward to working on such a study in the future with better anthropometric tools and its surgical validation.

## Conclusions

We observed in our study that there is a definite mathematical relationship between the length of the abdomen and the waist position, which may be applied for female waist sculpting.

## References

[1] Harper M, Lassetter J (2019). Cryolipolysis: a guide for primary care practitioners. J Nurse Pract.

[2] Lee NY, Robinson DM (2017). Noninvasive body contouring. Semin Cutan Med Surg.

[3] Lee SJ, Garg S, Lee HP (2014). Computer-aided analysis of the "beautiful" umbilicus. Aesthet Surg J.

[4] Stoff A, Richter DF (2015). Abdominoplasty and body contouring. Plastic and Reconstructive Surgery.

[5] Richter DF, Stoff A (2011). The scarpa lift--a novel technique for minimal invasive medial thigh lifts. Obes Surg.

[6] Richter DF, Stoff A, Velasco-Laguardia FJ, Reichenberger MA (2008). Circumferential lower truncal dermatolipectomy. Clin Plast Surg.

[7] Richter DF, Stoff A (2014). Circumferential body contouring: the lower body lift. Clin Plast Surg.

[8] Saldanha OR, Federico R, Daher PF (2009). Lipoabdominoplasty. Plast Reconstr Surg.

[9] Wu F (1998). The Poetics of Decadence: Chinese Poetry of the Southern Dynasties and Late Tang Periods. SUNY Press.

[10] Guerra RS, Amaral TF, Marques EA, Mota J, Restivo MT (2012). Anatomical location for waist circumference measurement in older adults: a preliminary study. Nutr Hosp.

[11] Veitch D (2012). Where is the human waist? Definitions, manual compared to scanner measurements. Work.

[12] Teimourian B, Adham MN, Malekzadeh S (1998). Waistline cincture. Aesthet Surg J.

